This article has been retracted.

# SARS–CoV–2 Spike Impairs DNA Damage Repair and Inhibits V(D)J Recombination In Vitro

**DOI:** 10.3390/v13102056

**Published:** 2021-10-13

**Authors:** Hui Jiang, Ya-Fang Mei

**Affiliations:** 1 Department of Molecular Biosciences, The Wenner–Gren Institute, Stockholm University, SE-10691 Stockholm, Sweden; 2 Department of Clinical Microbiology, Virology, Umeå University, SE-90185 Umeå, Sweden

**Keywords:** SARS–CoV–2, spike, DNA damage repair, V(D)J recombination, vaccine

## Abstract

Severe acute respiratory syndrome coronavirus 2 (SARS–CoV–2) has led to the coronavirus disease 2019 (COVID–19) pandemic, severely affecting public health and the global economy. Adaptive immunity plays a crucial role in fighting against SARS–CoV–2 infection and directly influences the clinical outcomes of patients. Clinical studies have indicated that patients with severe COVID–19 exhibit delayed and weak adaptive immune responses; however, the mechanism by which SARS–CoV–2 impedes adaptive immunity remains unclear. Here, by using an in vitro cell line, we report that the SARS–CoV–2 spike protein significantly inhibits DNA damage repair, which is required for effective V(D)J recombination in adaptive immunity. Mechanistically, we found that the spike protein localizes in the nucleus and inhibits DNA damage repair by impeding key DNA repair protein BRCA1 and 53BP1 recruitment to the damage site. Our findings reveal a potential molecular mechanism by which the spike protein might impede adaptive immunity and underscore the potential side effects of full-length spike-based vaccines.

## 1. Introduction

Severe acute respiratory syndrome coronavirus 2 (SARS–CoV–2) is responsible for the ongoing coronavirus disease 2019 (COVID–19) pandemic that has resulted in more than 2.3 million deaths. SARS–CoV–2 is an enveloped single positive–sense RNA virus that consists of structural and non–structural proteins [1]. After infection, these viral proteins hijack and dysregulate the host cellular machinery to replicate, assemble, and spread progeny viruses [2]. Recent clinical studies have shown that SARS–CoV–2 infection extraordinarily affects lymphocyte number and function [3,4,5,6]. Compared with mild and moderate survivors, patients with severe COVID–19 manifest a significantly lower number of total T cells, helper T cells, and suppressor T cells [3,4]. Additionally, COVID–19 delays IgG and IgM levels after symptom onset [5,6]. Collectively, these clinical observations suggest that SARS–CoV–2 affects the adaptive immune system. However, the mechanism by which SARS–CoV–2 suppresses adaptive immunity remains unclear. 

As two critical host surveillance systems, the immune and DNA repair systems are the primary systems that higher organisms rely on for defense against diverse threats and tissue homeostasis. Emerging evidence indicates that these two systems are interdependent, especially during lymphocyte development and maturation [7]. As one of the major double-strand DNA break (DSB) repair pathways, non-homologous end joining (NHEJ) repair plays a critical role in lymphocyte–specific recombination–activating gene endonuclease (RAG) –mediated V(D)J recombination, which results in a highly diverse repertoire of antibodies in B cell and T cell receptors (TCRs) in T cells [8]. For example, loss of function of key DNA repair proteins such as ATM, DNA–PKcs, 53BP1, et al., leads to defects in the NHEJ repair which inhibit the production of functional B and T cells, leading to immunodeficiency [7,9,10,11]. In contrast, viral infection usually induces DNA damage via different mechanisms, such as inducing reactive oxygen species (ROS) production and host cell replication stress [12,13,14]. If DNA damage cannot be properly repaired, it will contribute to the amplification of viral infection-induced pathology. Therefore, we aimed to investigate whether SARS–CoV–2 proteins hijack the DNA damage repair system, thereby affecting adaptive immunity in vitro. 

## 2. Materials and Methods

### 2.1. Antibodies and Reagents

DAPI (Cat #MBD0015), doxorubicin (Cat #D1515), H_2_O_2_ (Cat #H1009), and β-tubulin antibodies (Cat #T4026) were purchased from Sigma-Aldrich. Antibodies against His tag (Cat #12698), H2A (Cat #12349), H2A.X (Cat #7631), γ–H2A.X (Cat #2577), Ku80 (Cat # 2753), and Rad51(Cat #8875) were purchased from Cell Signaling Technology (Danvers, MA, USA). 53BP1(Cat #NB100-304) and RNF168 (Cat #H00165918–M01) antibodies were obtained from Novus Biologicals (Novus Biologicals, Littleton, CO, USA). Lamin B (Cat #sc–374015), ATM (Cat #sc–135663), DNA–PK (Cat #sc–5282), and BRCA1(Cat #sc–28383) antibodies were purchased from Santa Cruz Biotechnology (Santa Cruz, CA, USA). XRCC4 (Cat #PA5–82264) antibody was purchased from Thermo Fisher Scientific (Waltham, MA, USA).

### 2.2. Plasmids

pHPRT–DRGFP and pCBASceI were kindly gifted by Maria Jasin (Addgene plasmids #26476 and #26477) [15]. pimEJ5GFP was a gift from Jeremy Stark (Addgene plasmid #44026) [16]. The NSP1, NSP9, NSP13, NSP14, NSP16, spike, and nucleocapsid proteins were first synthesized with codon optimization and then cloned into a mammalian expression vector pUC57 with a C–terminal 6xHis tag. A 12–spacer RSS–GFP inverted complementary sequence–a 23–spacer RSS was synthesized for the V(D)J reporter vector. Then, the sequence was cloned into the pBabe–IRES–mRFP vector to generate the pBabe–12RSS–GFPi–23RSS–IRES–mRFP reporter vector. 12–spacer RSS sequence: 5′–CACAGTGCTACAGACTGGAACAAAAACC–3′. 23–spacer RSS sequence: 5′–CACAGTGGTAGTACTCCACTGTCTGGCTGTACAAAAACC–3′. RAG1 and RAG2 expression constructs were generously gifted by Martin Gellert (Addgene plasmid #13328 and #13329) [17].

### 2.3. Cells and Cell Culture 

HEK293T and HEK293 cells obtained from the American Type Culture Collection (ATCC) were cultured under 5% CO_2_ at 37 °C in Dulbecco’s modified Eagle’s medium (DMEM, high glucose, GlutaMAX) (Life Technologies, Carlsbad, CA, USA) containing 10% (*v*/*v*) fetal calf serum (FCS, Gibco), 1% (*v*/*v*) penicillin (100 IU/mL), and streptomycin (100 μg/mL). HEK293T–DR–GFP and HEK293T–EJ5–GFP reporter cells were generated as previously described and cultured under 5% CO_2_ at 37 °C in the above-mentioned culture medium.

### 2.4. HR and NHEJ Reporter Assays

HR and NHEJ repair in HEK293T cells were measured as described previously using DR–GFP and EJ5–GFP stable cells. Briefly, 0.5 × 10^6^ HEK293T stable reporter cells were seeded in 6–well plates and transfected with 2 μg I–SceI expression plasmid (pCBASceI) together with SARS–CoV–2 proteins expression plasmids. Forty–eight hours post–transfection and aspirin treatment, cells were harvested and analyzed by flow cytometry analysis for GFP expression. The means were obtained from three independent experiments.

### 2.5. Cellular Fractionation and Immunoblotting

For the cellular fraction assay, the Subcellular Protein Fractionation Kit (Thermo Fisher) was used according to the manufacturer’s instructions. Protein lysates were quantified using the BCA reagent (Thermo Fisher Scientific, Rockford, IL, USA). Proteins were resolved by sodium dodecyl sulfate–polyacrylamide gel electrophoresis (SDS–PAGE), transferred to nitrocellulose membranes (Amersham protran, 0.45 μm NC), and immunoblotted with specific primary antibodies followed by HRP–conjugated secondary antibodies. Protein bands were detected using SuperSignal West Pico or Femto Chemiluminescence kit (Thermo Fisher Scientific). 

### 2.6. Comet Assay

Cells were treated with different DNA damage reagents and then harvested at the indicated time points for analysis. Cells (1 × 10^5^ cells/mL in cold phosphate-buffered saline [PBS]) were resuspended in 1% low–melting agarose at 40 °C at a ratio of 1:3 vol/vol and pipetted onto a CometSlide. Slides were then immersed in prechilled lysis buffer (1.2 M NaCl, 100 mM EDTA, 0.1% sodium lauryl sarcosinate, 0.26 M NaOH pH > 13) for overnight (18–20 h) lysis at 4 °C in the dark. Slides were then carefully removed and submerged in rinse buffer (0.03 M NaOH and 2 mM EDTA, pH > 12) at room temperature (RT) for 20 min in the dark. This washing step was repeated twice. The slides were transferred to a horizontal electrophoresis chamber containing rinse buffer and separated for 25 min at a voltage of 0.6 V/cm. Finally, the slides were washed with distilled water, stained with 10 μg/mL propidium iodide, and analyzed by fluorescence microscopy. Twenty fields with approximately 100 cells in each sample were evaluated and quantified using the Fiji software to determine the tail length (tail moment). 

### 2.7. Immunofluorescence

Cells were seeded on glass coverslips in a 12–well plate and transfected with the indicated plasmid for 24 h. Then, the cells were treated with or without DNA damage reagents according to the experimental setup. The cells were fixed in 4% paraformaldehyde (PFA) in PBS for 20 min at RT and then permeabilized in 0.5% Triton X–100 for 10 min. Slides were blocked in 5% normal goat serum (NGS) and incubated with primary antibodies diluted in 1% NGS overnight at 4 °C. Samples were then incubated with the indicated secondary antibodies labeled with Alexa Fluor 488 or 555 (Invitrogen) diluted in 1% NGS at RT for 1 h. Thereafter, they were stained with DAPI for 15 min at RT. Coverslips were mounted using Dako Fluorescence Mounting Medium (Agilent) and imaged using a Nikon confocal microscope (Eclipse C1 Plus). All scoring was performed under blinded conditions. 

### 2.8. Analysis of V(D)J Recombination

Briefly, V(D)J reporter plasmid contains inverted-GFP and IRES driving continuously expressed RFP. Continuously expressed RFP is the internal transfection control. After Recombination activation gene1/2 (RAG1/2) co–transfected into the cells, RAG1/2 will cut the RSS and mediated induction of DSBs, if V(D)J recombination occurs, the inverted GFPs are ligated in positive order by NHEJ repair. Then the cell will express functional GFP. So, the GFP and RFP double positive cells are the readout of the V(D)J reporter assay [18]. 293T cells at 70% confluency were transfected with the V(D)J GFP reporter alone (background) or in combination with RAG1 and RAG2 expression constructs, at a ratio of 1 µg V(D)J GFP reporter: 0.5 µg RAG1: 0.5 µg RAG2. The following day, the medium was changed, and after an additional 48 h, cells were harvested and analyzed by flow cytometry for GFP and RFP expression.

### 2.9. Statistical Analysis

All experiments were repeated at least three times using independently collected or prepared samples. Data were analyzed by Student’s t test or ANOVA followed by Tukey’s multiple-comparison tests using GraphPad 8.

## 3. Results

### 3.1. Effect of Nuclear–Localized SARS–CoV–2 Viral Proteins on DNA Damage Repair 

DNA damage repair occurs mainly in the nucleus to ensure genome stability. Although SARS–CoV–2 proteins are synthesized in the cytosol [1], some viral proteins are also detectable in the nucleus, including Nsp1, Nsp5, Nsp9, Nsp13, Nsp14, and Nsp16 [19]. We investigated whether these nuclear-localized SARS–CoV–2 proteins affect the host cell DNA damage repair system. For this, we constructed these viral protein expression plasmids together with spike and nucleoprotein expression plasmids, which are generally considered cytosol–localized proteins. We confirmed their expression and localization by immunoblotting and immunofluorescence (Figure 1A and Figure S1A). Our results were consistent with those from previous studies [19]; Nsp1, Nsp5, Nsp9, Nsp13, Nsp14, and Nsp16 proteins are indeed localized in the nucleus, and nucleoproteins are mainly localized in the cytosol. Surprisingly, we found the abundance of the spike protein in the nucleus (Figure 1A). NHEJ repair and homologous recombination (HR) repair are two major DNA repair pathways that not only continuously monitor and ensure genome integrity but are also vital for adaptive immune cell functions [9]. To evaluate whether these viral proteins impede the DSB repair pathway, we examined the repair of a site-specific DSB induced by the I–SceI endonuclease using the direct repeat–green fluorescence protein (DR–GFP) and the total-NHEJ-GFP (EJ5–GFP) reporter systems for HR and NHEJ, respectively [15,16]. Overexpression of Nsp1, Nsp5, Nsp13, Nsp14, and spike proteins diminished the efficiencies of both HR and NHEJ repair (Figure 1B–E and Figure S2A,B). Moreover, we also found that Nsp1, Nsp5, Nsp13, and Nsp14 overexpression dramatically suppressed proliferation compared with other studied proteins (Figure S3A,B). Therefore, the inhibitory effect of Nsp1, Nsp5, Nsp13, and Nsp14 on DNA damage repair may be due to secondary effects, such as growth arrest and cell death. Interestingly, overexpressed spike protein did not affect cell morphology or proliferation but significantly suppressed both HR and NHEJ repair (Figure 1B–E, Figures S2A,B and S3A,B). 

### 3.2. SARS–CoV–2 Spike Protein Inhibits DNA Damage Repair

Because spike proteins are critical for mediating viral entry into host cells and are the focus of most vaccine strategies [20,21], we further investigated the role of spike proteins in DNA damage repair and its associated V(D)J recombination. Spike proteins are usually thought to be synthesized on the rough endoplasmic reticulum (ER) [1]. After posttranslational modifications such as glycosylation, spike proteins traffic via the cellular membrane apparatus together with other viral proteins to form the mature virion [1]. Spike protein contains two major subunits, S1 and S2, as well as several functional domains or repeats [22] (Figure 2A). In the native state, spike proteins exist as inactive full–length proteins. During viral infection, host cell proteases such as furin protease activate the S protein by cleaving it into S1 and S2 subunits, which is necessary for viral entry into the target cell [23]. We further explored different subunits of the spike protein to elucidate the functional features required for DNA repair inhibition. Only the full–length spike protein strongly inhibited both NHEJ and HR repair (Figure 2B–E and Figure S4A,B). Next, we sought to determine whether the spike protein directly contributes to genomic instability by inhibiting DSB repair. We monitored the levels of DSBs using comet assays. Following different DNA damage treatments, such as γ–irradiation, doxorubicin treatment, and H_2_O_2_ treatment, there is less repair in the presence of the spike protein (Figure 2F,G). Together, these data demonstrate that the spike protein directly affects DNA repair in the nucleus.

### 3.3. Spike Proteins Impede the Recruitment of DNA Damage Repair Checkpoint Proteins

To confirm the existence of spike protein in the nucleus, we performed subcellular fraction analysis and found that spike proteins are not only enriched in the cellular membrane fraction but are also abundant in the nuclear fraction, with detectable expression even in the chromatin–bound fraction (Figure 3A). We also observed that the spike has three different forms, the higher band is a highly glycosylated spike, the middle one is a full–length spike, and the lower one is a cleaved spike subunit. Consistent with the comet assay, we also found the upregulation of the DNA damage marker, γ–H2A.X, in spike protein–overexpressed cells under DNA damage conditions (Figure 3B). A recent study suggested that spike proteins induce ER stress and ER–associated protein degradation [24]. To exclude the possibility that the spike protein inhibits DNA repair by promoting DNA repair protein degradation, we checked the expression of some essential DNA repair proteins in NHEJ and HR repair pathways and found that these DNA repair proteins were stable after spike protein overexpression (Figure 3C). To determine how the spike protein inhibits both NHEJ and HR repair pathways, we analyzed the recruitment of BRCA1 and 53BP1, which are the key checkpoint proteins for HR and NHEJ repair, respectively. We found that the spike protein markedly inhibited both BRCA1 and 53BP1 foci formation (Figure 3D–G). Together, these data show that the SARS–CoV–2 full–length spike protein inhibits DNA damage repair by hindering DNA repair protein recruitment. 

### 3.4. Spike Protein Impairs V(D)J Recombination In vitro

DNA damage repair, especially NHEJ repair, is essential for V(D)J recombination, which lies at the core of B and T cell immunity [9]. To date, many approved SARS–CoV–2 vaccines, such as mRNA vaccines and adenovirus–COVID–19 vaccines, have been developed based on the full–length spike protein [25]. Although it is debatable whether SARS–CoV–2 directly infects lymphocyte precursors [26,27], some reports have shown that infected cells secrete exosomes that can deliver SARS–CoV–2 RNA or protein to target cells [28,29]. We further tested whether the spike protein reduced NHEJ–mediated V(D)J recombination. For this, we designed an in vitro V(D)J recombination reporter system according to a previous study [18] (Figure S5). Compared with the empty vector, spike protein overexpression inhibited RAG–mediated V(D)J recombination in this in vitro reporter system (Figure 4). 

## 4. Discussion

Our findings provide evidence of the spike protein hijacking the DNA damage repair machinery and adaptive immune machinery in vitro. We propose a potential mechanism by which spike proteins may impair adaptive immunity by inhibiting DNA damage repair. Although no evidence has been published that SARS–CoV–2 can infect thymocytes or bone marrow lymphoid cells, our in vitro V(D)J reporter assay shows that the spike protein intensely impeded V(D)J recombination. Consistent with our results, clinical observations also show that the risk of severe illness or death with COVID–19 increases with age, especially older adults who are at the highest risk [22]. This may be because SARS–CoV–2 spike proteins can weaken the DNA repair system of older people and consequently impede V(D)J recombination and adaptive immunity. In contrast, our data provide valuable details on the involvement of spike protein subunits in DNA damage repair, indicating that full–length spike–based vaccines may inhibit the recombination of V(D)J in B cells, which is also consistent with a recent study that a full–length spike–based vaccine induced lower antibody titers compared to the RBD–based vaccine [28]. This suggests that the use of antigenic epitopes of the spike as a SARS–CoV–2 vaccine might be safer and more efficacious than the full–length spike. Taken together, we identified one of the potentially important mechanisms of SARS–CoV–2 suppression of the host adaptive immune machinery. Furthermore, our findings also imply a potential side effect of the full–length spike–based vaccine. This work will improve the understanding of COVID–19 pathogenesis and provide new strategies for designing more efficient and safer vaccines. 

## Figures and Tables

**Figure 1:** Effect of severe acute respiratory syndrome coronavirus 2 (SARS–CoV–2) nuclear-localized proteins on DNA damage repair. (**A**) Subcellular distribution of the SARS–CoV–2 proteins. Immunofluorescence was performed at 24 h after transfection of the plasmid expressing the viral proteins into HEK293T cells. Scale bar: 10 µm. (**B**) Schematic of the EJ5-GFP reporter used to monitor non-homologous end joining (NHEJ). (**C**) Effect of empty vector (E.V) and SARS–CoV–2 proteins on NHEJ DNA repair. The values represent the mean ± standard deviation (SD) from three independent experiments (see representative FACS plots in Figure S2A). (**D**) Schematic of the DR-GFP reporter used to monitor homologous recombination (HR). (**E**) Effect of E.V and SARS–CoV–2 proteins on HR DNA repair. The values represent the mean ± SD from three independent experiments (see representative FACS plots in Figure S2B). The values represent the mean ± SD, *n* = 3. Statistical significance was determined using one-way analysis of variance (ANOVA) in (**C**,**E**). ** *p* < 0.01, *** *p* < 0.001, **** *p* <  0.0001.

**Figure 2:** Severe acute respiratory syndrome coronavirus 2 (SARS–CoV–2) spike protein inhibits DNA damage repair. (**A**) Schematic of the primary structure of the SARS–CoV–2 spike protein. The S1 subunit includes an N–terminal domain (NTD, 14–305 residues) and a receptor–binding domain (RBD, 319–541 residues). The S2 subunit consists of the fusion peptide (FP, 788–806 residues), heptapeptide repeat sequence 1 (HR1, 912–984 residues), HR2 (1163–1213 residues), TM domain (TM, 1213–1237 residues), and cytoplasm domain (CT,1237–1273 residues). (**B**,**C**) Effect of titrated expression of the spike protein on DNA repair in HEK–293T cells. (**D**,**E**) Only full-length spike protein inhibits non-homologous end joining (NHEJ) and homologous recombination (HR) DNA repair. The values represent the mean ± SD from three independent experiments (see representative FACS plots in Figure S4A,B). (**F**) Full–length spike (S–FL) protein–transfected HEK293T cells exhibited more DNA damage than empty vector-, S1–, and S2–transfected cells under different DNA damage conditions. For doxorubicin: 4 µg/mL, 2 h. For γ–irradiation: 10 Gy, 30 min. For H_2_O_2_: 100 µM, 1 h. Scale bar: 50 µm. (**G**) Corresponding quantification of the comet tail moments from 20 different fields with *n* > 200 comets of three independent experiments. Statistical significance was assessed using a two-way analysis of variance (ANOVA). NS (Not Significant): * *p* > 0.05, ** *p* < 0.01, *** *p* < 0.001, **** *p* < 0.0001.

**Figure 3:** Severe acute respiratory syndrome coronavirus 2 (SARS–CoV–2) spike protein impedes the recruitment of DNA damage repair checkpoint proteins. (**A**) Membrane fraction (MF), cytosolic fraction (CF), soluble nuclear fraction (SNF), and chromatin-bound fraction (CBF) from HEK293T cells transfected with SARS–CoV–2 spike protein were immunoblotted for His-tag spike and indicated proteins. (**B**) Left: Immunoblots of DNA damage marker γH2AX in empty vector (E.V)– and spike protein–expressing HEK293T cells after 10 Gy γ-irradiation. Right: corresponding quantification of immunoblots in left. The values represent the mean ± SD (*n* = 3). Statistical significance was determined using Student’s *t*-test. **** *p* < 0.0001. (**C**) Immunoblots of DNA damage repair related proteins in spike protein–expressing HEK293T cells. (**D**) Representative images of 53BP1 foci formation in E.V– and spike protein-expressing HEK293 cells exposed to 10 Gy γ–irradiation. Scale bar: 10 µm. (**E**) Quantitative analysis of 53BP1 foci per nucleus. The values represent the mean ± SEM, *n* = 50. (**F**) BRCA1 foci formation in empty vector- and spike protein-expressing HEK293 cells exposed to 10 Gy γ–irradiation. Scale bar: 10 µm. (**G**). Quantitative analysis of BRCA1 foci per nucleus. The values represent the mean ± SEM, *n* = 50. Statistical significance was determined using Student’s *t*-test. **** *p* < 0.0001.

**Figure 4:** Spike protein impairs V(D)J recombination in vitro. (**A**) Schematic of the V(D)J reporter system. (**B**) Representative plots of flow cytometry show that the SARS–CoV–2 spike protein impedes V(D)J recombination in vitro. (**C**) Quantitative analysis of relative V(D)J recombination. The values represent the mean ± SD, *n* = 3. Statistical significance was determined using Student’s *t*-test. **** *p* < 0.0001.

## Data Availability

The data presented in this study are available in the main text and Supplementary Materials.

## Supplementary Materials

The following are available online at https://www.mdpi.com/article/10.3390/v13102056/s1, Figure S1: Expression of nuclear–localized SARS–CoV–2 proteins in human cells, Figure S2: Effect of nuclear SARS–CoV–2 proteins on NHEJ– and HR–DNA repair pathway, Figure S3: Nsp1, Nsp5, Nsp13, Nsp14 but not spike inhibit cell proliferation, Figure S4: Effect of SARS–CoV–2 spike mutants on NHEJ– and HR– DNA repair pathway, Figure S5: In vitro V(D)J recombination assay.
